# Protective Effect of Keluoxin against Diabetic Nephropathy in Type 2 Diabetic Mellitus Models

**DOI:** 10.1155/2021/8455709

**Published:** 2021-10-19

**Authors:** Xiaomei Yang, Xuke Han, Qing Wen, Xianliang Qiu, Huan Deng, Qiu Chen

**Affiliations:** ^1^School of Clinical Medicine, Chengdu University of Traditional Chinese Medicine, Chengdu 610075, China; ^2^Department of Endocrinology, Hospital of Chengdu University of Traditional Chinese Medicine, Chengdu 610072, China

## Abstract

Diabetic nephropathy (DN) is a chronic kidney disease that develops in patients with diabetes mellitus (DM). Renal dysfunction and persistent proteinuria are the main clinical features of DN. Podocyte injury is an important cause of persistent proteinuria and diabetic kidney disease (DKD) progression. Traditional Chinese patent medicines can improve renal function by enhancing autophagy and promoting apoptosis. Keluoxin is a Chinese patent medicine that has the effect of invigorating qi and nourishing yin, activating blood, and eliminating blood stasis. Therefore, we hypothesized that Keluoxin may have a protective effect against diabetic nephropathy in rats with type 2 DM. Rats induced with diabetes through streptozocin (STZ) injection and a high-fat and high-sugar diet were treated with Keluoxin (0.63 g/kg/day) for 8 weeks, and renal function, biochemical indicators, and histopathological changes in renal tissues were observed. Immunofluorescence staining and western blot analysis were used to detect the expression of autophagy-related proteins. The results showed that Keluoxin reduced blood glucose and lipid levels, improved renal function, and alleviated renal histopathological changes in rats with DN. The therapeutic effect was similar to that of Irbesartan (15.6 mg/kg/day). It is inferred that the mechanism works through reducing the obstruction of downstream pathways of autophagy by improving the lysosomal degradation function and alleviating podocyte injury. This study demonstrates that Keluoxin could regulate autophagy in podocytes, alleviate kidney injury in rats with DN, and have a protective effect on renal function; its mechanism can thus be a potential therapy for DN.

## 1. Introduction

Diabetic nephropathy (DN) is one of the most common microvascular complications in diabetes mellitus (DM); it has become the main cause of chronic kidney disease (CKD) in developed countries and is an important cause of end-stage nephropathy in China [1, 2]. The study found that the prevalence of diabetic kidney disease (DKD) in the Chinese diabetic population is approximately 20–40%, which seriously affects the quality of life of patients [3]. The causes of DN are complicated; however, a study has shown that podocyte injury is an important cause of proteinuria persistence and DKD progression [4]. Podocytes are epithelial cells of the glomerular visceral layer and are highly specialized, terminally differentiated cells that attach themselves to the lateral basement membrane of the glomerulus, which is an important part of the glomerular filtration barrier [5]. Recent studies have established that glomerular podocytes are damaged in the early stage of diabetes; podocyte injury is closely related to the occurrence and development of DKD and is the core factor in DKD progression [6]. Although podocytes are crucial for the development of DN, the mechanism of podocyte injury has not been well elucidated.

Autophagy of cells may be the pathological basis of DN and has been widely studied in recent years [7]. It is a lysosome-dependent protein degradation pathway that regulates cellular homeostasis and metabolism under stress conditions [8, 9]. Autophagy plays a key role in maintaining the structure and function of podocytes, and its excessive activation or inhibition is the cause of podocyte damage [4]. Studies have shown that autophagy imbalance alters podocyte structure and function in patients with DM, and impaired autophagy, damaged podocytes, and massive proteinuria were observed in diabetic patients or rats induced with diabetes [10, 11]. Thus, autophagy plays an important role in human health and diseases, including kidney injury [12, 13]. Growing evidence suggests that impairment of renal autophagy is involved in the pathogenesis of DN and that recovery of autophagy may be the key to renal protection [7, 14]. Protein 1 light chain 3B (LC3) and p62 are autophagy-related proteins, and studies have shown that persistent high glucose (HG) in DN leads to increased activation of renal epidermal growth factor receptor (EGFR) signals, inhibits autophagy-associated protein expression, and decreases autophagy activity [10, 15]. Impaired autophagy activity contributes to the pathogenesis of DN. Therefore, recovery of autophagy activity may be a promising therapy for DN [16, 17].

Traditional Chinese medicine, for example, Rhizoma Coptidis, Curcumin, Yishen capsule, Celastrol, and Hirudin, has achieved remarkable results in the treatment of DN [2, 18–21]. Keluoxin is a Chinese patent medicine that has the function of raising yin, activating blood, and eliminating blood stasis. Its drug composition includes Astragalus, Radix Pseudostellariae, *Lycium barbarum*, *Ligustrum lucidum*, Leech, and Rhubarb, which are mainly used in the treatment of qi and yin deficiency and blood stasis in diabetes. Studies have shown that *Astragalus membranaceus*, Rhubarb, and Hirudin can reduce glomerular pathological changes by regulating autophagy and reduce mean blood glucose level, body weight, urinary albumin excretion, and serum creatinine level in rats with DN, thereby improving renal function [22–26]. Ginsenoside Rg1 significantly alleviates renal fibrosis and podocyte epithelial-mesenchymal transition (EMT) in diabetic rats and podocytes exposed to high glucose levels [9]. *Ligustrum lucidum*, Radix Pseudostellariae, and Lycium medlar also have certain protective effects on renal function and can reduce damage to DN podocytes. A study showed that Chinese patent medicine with the Yiqi Yangyin Huayu formula can reduce the level of urinary protein, reverse renal ultrastructural changes in rats with DN, alleviate the early onset of DN, and inhibit its progression [27]. Chinese patent medicine thus plays an important role in the treatment and delaying of DN. Based on these facts, we hypothesized that Keluoxin may have a protective effect against DN in type 2 DM patients. The aim of this study is to determine the protective effect of Keluoxin against DN in a model of type 2 DM.

## 2. Materials and Methods

### 2.1. Experimental Animals

Male Sprague Dawley rats weighing 200 ± 20 g (*n* = 28) were sourced from the Chengdu Dossy Experimental Animals Company. All rats were housed in a specific pathogen-free (SPF) animal room, maintained at 24 ± 1°C with a regular 12 h light/dark cycle, and granted free access to water and food for one week before starting the experiment. The standard laboratory chow and tap water were available ad libitum. All animal experimental protocols were based on international guidelines and approved by the Ethics Committee of Chengdu Dossy Experimental Animals Company.

### 2.2. Induction and Treatment of Type 2 Diabetic Nephropathy

Seven rats were randomly selected to form the normal group, and the remaining 21 rats were used to establish the model. The rats in the normal group received a normal diet, while the other 21 rats received a high-fat, high-sugar diet. The right kidneys of the rats were surgically removed after 4 weeks of feeding. Two weeks after the surgery, streptozocin (STZ, 40 mg/kg) was intraperitoneally injected into the 21 rats in the experimental group, and the normal group was injected with the same volume of saline (pH = 4.5); after 72 h, fasting blood glucose levels were determined using blood samples from the tail vein, in all the rats. Rats with a serum glucose level ≥16.7 mmol/L for three consecutive days were deemed as representing the DM model. After two weeks, the urine over a 24 h period of rats in the experimental group was collected, and their urine microalbumin levels were found to be greater than 30 mg/24 h; the DN model in rats was thus successfully created. The rats representing the model were then randomly divided into three groups: the DN group (model group), Keluoxin group (Keluoxin purchased from Chengdu Kanghong Pharmaceutical Company, 1911002), and Irbesartan group (Irbesartan purchased from Shanghai Yuanye Bio-Technology Company, S27F8D30066), with seven rats in each group. Rats in the normal group and model group were administered with normal saline (10 ml/kg/day), while those in the Keluoxin group were treated with Keluoxin suspension prepared from capsules (0.63 g/kg/day), and those in the Irbesartan group were treated with Irbesartan (15.6 mg/kg/day). Rats in all the groups were observed for eight weeks. Eight weeks later, the rats were sacrificed.

### 2.3. Determination of Biochemical Indices

Spot urine and serum samples were collected just before euthanasia. Blood samples were collected from the abdominal aorta of rats under mild ether anesthesia in heparinized centrifuge tubes. The samples were immediately centrifuged at 3500 rpm to separate the plasma, extract the supernatant, and determine the relevant indicators. The appropriate kits purchased from Abcam (Cambridge, MA, USA) were used to measure fasting plasma glucose (FPG), 2 h oral glucose tolerance test (2 h OGTT) values, total cholesterol (TC), glycerin trilaurate (TG), high-density lipoprotein cholesterol (HDL-C), and low-density lipoprotein cholesterol (LDL-C). Commercial kits purchased from Bethyl Laboratories (Montgomery, AL, USA) were used to measure urine microalbumin (MAU), uric creatinine (UCr), the ratio of urine microalbumin/uric creatinine, urea, and serum creatinine (SCr) levels in rats.

### 2.4. Histopathological Examination

The renal tissues were fixed with 10% neutral formaldehyde, dehydrated using alcohol, embedded in paraffin, cut into 6 *μ*m sections, and stained with hematoxylin-eosin (HE), periodic acid-Schiff (PAS), and Masson. Then, all sections were observed and photographed through light microscopy. The rest of the renal tissue was frozen in liquid nitrogen at −80°C for western blot detection. After HE staining treatment, the degree of tubular stromal damage was assessed by semiquantitative, with scoring criteria being 0 (no damage), 1 (≤10%), 2 (11%∼25%), 3 (26%∼45%), 4 (46%∼75%), and 5 (>76%). At least 10 choroid boundary fields were selected for each section. The positive expression area percentage (% area) and the light density (integrated optical density, IOD) were measured using the Image J-win64 image analysis system, and the percentage of the expression area in the fiber tissue was calculated; the statistical analysis software SPSS 22.0 was applied to perform single factor variance analysis (one-way ANOVA) on the data, the variance represented by mean ± standard difference (*x* ± SD).

### 2.5. Immunofluorescence Staining

Renal tissues were embedded in optimum cutting temperature compounds by snap freezing in liquid nitrogen. The frozen sections (6 *μ*m) were fixed with cold acetone for 10 min, blocked in PBS containing 10% goat serum at room temperature for 30 min, and incubated with primary antibodies against nephrin at 4°C overnight. After several PBS rinses, CyTM 2-conjugated secondary antibodies were applied for 30 min at room temperature. The nuclei were visualized using 4,6-diamidino-2-phenylindole (DAPI) staining. After several PBS rinses, the sections were mounted with an antiflu-fluorescent attenuating agent. Images were recorded using a Leica laser scanning microscope (Leica DM IRB, Leica, Wetzlar, Germany). The fluorescence intensity (intDen) and area (Area) of all the collected images were measured, and the average fluorescence intensity (mean) of each image was calculated using the Image J-win64 image analysis system; the statistical analysis software SPSS 22.0 was applied to perform single factor variance analysis (one-way ANOVA) on the data. The results of the statistical analyses were represented by mean ± standard difference (*x* ± SD).

### 2.6. Western Blot Analysis

Renal cortical tissues were collected and frozen at −80°C. The concentration of extracted protein was detected using the Protein BCA Assay (Beyotime, Jiangsu, China, Item number: P0009). Proteins were separated by 10% sodium dodecyl sulfate-polyacrylamide gel electrophoresis (Shanghai Yase Biotechnology Co., Ltd., No. PG112) and transferred onto nitrocellulose membranes (Sigma Aldrich, Goods No. ISEQ00010). After blocking with nonfat milk, primary antibodies specific for *β*-actin (Rabbit Clone antibody, cargo number: ab207612, Abcam-AbResistance (Shanghai) Trading Co., Ltd.), p62 (P62 Antibody, Rabbit Clone antibody, cargo number: ab91526, Abcam-AbResistance (Shanghai) Trading Co., Ltd), LC3B (rabbit clone antibody, cargo number: ab48394, Abcam-AbResistance (Shanghai) Trading Co., Ltd), and nephrin (Rabbit clonal antibody, cargo number: DF7501, affinity) were used. Goat anti-rabbit IgG conjugated with horseradish peroxidase was used to detect the expression of primary antibodies, and protein bands were visualized using an ECL western blotting detection system (Amersham, Little Chalfont, UK).

### 2.7. Statistical Analysis

SPSS 22.0 was used to analyze the experimental data. The measurement data were expressed as mean ± standard deviation (*X* ± SD). Data were compared by one-way ANOVA test, followed by the SNK-q test between different groups. If there was no special explanation, *P* < 0.05 was considered statistically significant.

## 3. Results

The following changes were observed in rats induced with DN after treatment with Keluoxin.

### 3.1. Changes in Renal Function

As shown in Table 1, compared with the normal group, the weight of rats in the model group showed a significant reduction (*P* < 0.01), and their urine volume showed a significant increase (*P* < 0.01). Compared with the model group, the urine volumes of rats in the Keluoxin and Irbesartan groups were significantly lower (*P* < 0.01); their weights were slightly less, but there were no significant differences compared with the model group. As shown in Figure 1, in the model group, the UREA, MAU, and the MAU/UCR ratio increased significantly (*P* < 0.01) and the SCr level decreased significantly (*P* < 0.01) compared with the normal group; UCr level did not change significantly, indicating early renal injury in rats with DN. Compared to the model group, the MAU and MAU/UCR ratios in the Keluoxin group were significantly lower (*P* < 0.01), while the decrease in UREA levels was not statistically significant. The MAU/UCR ratio in the Irbesartan group showed a significant reduction (*P* < 0.01), while the decreases in the levels of UREA and MAU were not statistically significant.

### 3.2. Changes in Biochemical Indices

As shown in Table 2, compared with the normal group, the TG levels in the model group were significantly higher (*P* < 0.05), and no significant changes in TC, LDL-C, and HDL-C were observed. Compared with the model group, the values of TC, TG, and LDL-C were lower in the Keluoxin and Irbesartan groups while those of HDL-C were higher, but the differences were not statistically significant. As shown in Table 3, compared with the normal group, the fasting blood glucose and 2 h OGTT values in the model group were significantly higher (*P* < 0.01). Compared with the model group, the fasting blood glucose was significantly lower in the Keluoxin group (*P* < 0.01) , and the 2 h OGTT blood glucose showed improvement in the Keluoxin group, but the difference was not statistically significant. There was no significant improvement in the fasting blood glucose levels in the Irbesartan group, and although the 2 h OGTT showed improvement in this group, the improvement was not statistically significant.

### 3.3. Pathological Changes in Renal Tissues

Histologically, as shown in Figure 2, the renal tissue membrane of rats in the normal group was complete with no connective hyperplasia and inflammatory exudation; it had complete glomerular structure, no capillary substrate membrane or matrix hyperplasia, intact renal tubules, and no parenchymal or inflammatory cell infiltration in the renal tubule structure, and it exhibited a small blue area in the renal interstitium. The renal tissue membrane of rats with DN was relatively complete, showing glomerular membrane hyperplasia, cystic wall hyperplasia, renal tubular dilation, and epithelial cells balloon-like changes. The lesion basically complied with the pathological changes of diabetic nephropathy, suggesting that the diabetic nephropathy model was basically successful but the degree of molding is relatively mild. The renal tubules were slightly dilated, with substantial collagen deposits in the glomerular and renal tubules, and the renal interstitium showed a large blue area, indicating severe renal fibrosis in the renal tissue of rats with DN. After treatment with Keluoxin and Irbesartan, the renal tissue membrane of rats in the normal group was complete with no connective hyperplasia and inflammatory exudation; the renal pathological changes were significantly reduced, glomerular sclerosis and collagen deposition were significantly improved, and the blue area in the renal tissue was significantly reduced. Additionally, as shown in Figure 2(b), the percentage of collagen expression in the model group was significantly higher than that in the normal group (*P* < 0.01). The percentage of area under collagen expression was lower in the Keluoxin and Irbesartan groups compared to the model group (*P* < 0.01). As shown in Figure 2(c), the percentage of positively expressed glomerular area in the model group was significantly higher than that in the normal group (*P* < 0.05). The percentages of the glomerular area with positive expression in the Keluoxin and Irbesartan groups were lower than that in the model group (*P* < 0.05). Taken together, it can be inferred that treatment with Keluoxin significantly improved the pathology and restored the glomerular structure of renal tissues.

### 3.4. Alteration of Autophagy-Related Proteins in Renal Tissues

As shown in Table 4, compared with the normal group, the levels of p62 and LC3-ll protein in the model group were significantly higher (*P* < 0.01) as was the ratio of LC3-ll/LC3-l (*P* < 0.05), while nephrin protein was significantly lower in the model group (*P* < 0.01). Compared with the model group, the levels of LC3-II protein in the Keluoxin and Irbesartan groups decreased significantly (*P* < 0.05), and the expression of nephrin protein was significantly upregulated (*P* < 0.01). The levels of p62 in the Keluoxin and Irbesartan groups decreased significantly (*P* < 0.05, *P* < 0.01). The nephrin of podocyte markers under immunofluorescence staining was downregulated in rats with DN, indicating impairment of the glomerular filtration barrier. In addition, treatment with Keluoxin and Irbesartan upregulated the expression of nephrin in the renal tissue (Figures 3(e) and 4). As shown in Figure 3(f), the nephrin protein content in renal tissue was significantly less in the model group compared to that in the normal group (*P* < 0.05). Compared with the model group, the nephrin protein content in the Keluoxin and Irbesartan groups was significantly higher (*P* < 0.05).

## 4. Discussion

DN is characterized by impairment of renal function and development of proteinuria; morphological and functional changes in podocytes are important reasons for the occurrence and development of DN [28–30]. Podocytes are highly differentiated glomerular epithelial cells that form the glomerular filtration barrier, and they cannot regenerate after injury [31]. The study found that podocyte injury in DN was caused by a variety of factors including mechanical stress, inflammatory stress, oxidative stress, TGF-*β*1 induction, activation of the renin-angiotensin-aldosterone system (RAAS), and advanced glycation end product (AGE) accumulation [32]. Podocytes exhibit high levels of basal autophagy under physiological conditions [33]. Persistent HG in DN can inhibit the expression of autophagy-related proteins, weaken autophagy, and lead to irreversible cell damage and dysfunction [34–36]. Studies have observed insufficient autophagy and podocyte loss in diabetic patients with massive proteinuria; at the same time, they also found podocyte loss and massive proteinuria in diabetic mice, suggesting that impaired podocyte autophagy is involved in the pathogenesis of severe podocyte injury, leading to massive proteinuria associated with DN [37]. This is consistent with our observations, where the model group was found to have large amounts of urinary protein, indicating impaired renal function. Nephrin is the main protein in the foot process junction of the glomerular membrane that prevents protein filtration, and changes in its expression can indirectly reflect podocyte injury [38]. In this study, we observed that the level of nephrin protein decreased significantly in the model group, while the urine protein level in the model group was significantly higher than that in the normal group. Moreover, histopathological examination of the kidney showed that the glomeruli of the model group prominently exhibited sclerosis, atrophy, irregular thickening of the glomerular basement membrane, and dilated renal tubules and that the basement membrane of renal tubules was thickened, indicating severe renal injury in the DN-model rats. This is consistent with previous observations [19]. After treatment with Keluoxin, the expression of the podocyte marker protein nephrin was increased, and renal histopathological parameters significantly improved, indicating that Keluoxin can prevent podocyte injury and alleviate DN symptoms.

Obstruction of any of the autophagy processes, including autophagy induction, autophagy vacuole and lysosome fusion, and lysosome degradation of the autophagy vacuole, will affect autophagy activity [39]. The lysosome is an organelle containing various hydrolases, whose main activity is the degradation of cell components and macromolecules; it is located at the end of the autophagy pathway. The mediated degradation system is an important step in autophagy degradation [40]. LC3 and p62 are autophagy-related proteins, and studies have shown that AGEs can increase the expression of LC3-II and p62 proteins. This leads to an increase in the number of autophagosomes and failure of lysosomal conversion in LC3-II or p62, indicating that the degradation of autophagic vacuoles is blocked and the autophagy activity is severely inhibited [33, 41]. In our study, we established a rat model of DN induced by STZ and high-fat and high-sugar diets and observed a significant increase in the expression of LC3-II (*P* < 0.01) in DN-model rats, indicating that HG induces autophagy in podocytes, which is consistent with previous reports [42]. This phenomenon may be due to a self-protective stress response. Podocytes maintain their function and homeostasis by increasing autophagy within a short period of time after HG stimulation [20]. The expression of p62 proteins increased significantly (*P* < 0.01), indicating that autophagy activity in podocytes was inhibited under high glucose conditions. This may have occurred due to lysosomal dysfunction, which leads to obstruction of the downstream pathways of the autophagy process. After treatment with Keluoxin and Irbesartan, the expression of LC3-II and p62 proteins decreased significantly, suggesting that obstruction of the downstream pathways of autophagy was reduced, and the autophagy activity of the podocytes was restored. Therefore, we were able to confirm the regulative effect of Keluoxin and Irbesartan on renal function in rats with DN.

Thus, Keluoxin can improve the autophagy function of podocytes, alleviate renal injury, and protect renal function in rats with DN. Interestingly, this study found that Keluoxin and Irbesartan had similar efficacies and could regulate kidney function as a whole in rats with DN; the side effects of traditional Chinese medicine are also low.

## 5. Conclusions

Keluoxin can effectively improve blood glucose and blood lipid levels and renal function in rat DN models, which were established by inducing DN in rats using STZ. Keluoxin can alleviate renal histopathological changes and delay DN progression, and it has a protective effect against DN in a model of type 2 DM. This effect may be achieved by regulating autophagy in podocytes; the mechanism may be a potential therapy for DN which needs further investigation.

The limitations of this study include shortage of time, energy, and research funds. The observation period of the study was short and the sample size was small. Moreover, the effect of Keluoxin on rats with DN was observed only in terms of its effects on the autophagy mechanism in podocytes, other pathological mechanisms should be undertaken in future studies, such as oxidative stress, inflammatory mechanisms, and PI3K/AKT/mTOR signaling pathways. In addition, the actual active components of Chinese medicine in the blood after metabolism in vivo are not exactly the same as those in the original medicine; treatment of podocytes in vitro with serum-containing Keluoxin needs to be undertaken in future studies. Thus, an increasing number of studies using larger samples are needed to confirm the improvement of autophagy in podocytes with Keluoxin. These limitations need to be addressed in future studies.

## Figures and Tables

**Figure 1:** Effect of Keluoxin and Irbesartan on renal function of DN-induced rats. (a) The level of UREA; (b) the level of SCr; (c) the level of MAU; (d) the level of UCr; (e) the ratio of MAU/UCr. ^*∗*^*P* < 0.05 and ^*∗∗*^*P* < 0.01 versus the normal group; ^#^*P* < 0.05 and ^##^*P* < 0.01 versus the model group.

**Figure 2:** Effect of Keluoxin on histomorphological changes of renal tissues in DN-induced rats. Renal tissues were observed by staining with H&E, Masson, and PAS; the magnification is ×400. (a) Injury score (HE staining). (b) Percentage of collagen expression area in renal tissue (Masson staining). (c) The ratio of glomerular positive expression area (%) (PAS staining).

**Figure 3:** Effect of Keluoxin and Irbesartan on LC3, p62, and nephrin proteins in renal tissues of DN-induced rats. (a) The levels of LC3, p62, and nephrin proteins from renal tissues were detected by western blot and normalized to *β*-actin. (b) The expression of LC3-II. (c) The ratio of LC3-ll/LC3-l. (d) The expression of p62. (e) The expression of nephrin protein. (f) Mean fluorescence intensity of nephrin was measured for each group. ^*∗*^*P* < 0.05 and ^*∗∗*^*P* < 0.01 versus the normal group; ^#^*P* < 0.05 and ^##^*P* < 0.01 versus the model group.

**Figure 4:** Representative images of immunofluorescence staining for nephrin and 4′,6-diamidino-2-phenylindole (DAPI) staining for nuclei. Scale bars, 20 *μ*m.

**Table 1:** Comparisons of body weight and urine volume in different groups after 8 weeks.

Group	*N*	Body weight (g)	Urine volume (ml)
Normal	7	548.50 ± 51.09	15.60 ± 7.50
Model	7	384.78 ± 33.12^*∗∗*^	139.86 ± 29.70^*∗∗*^
Keluoxin	7	341.93 ± 47.72^*∗∗*^	57.71 ± 36.52^*∗∗*##^
Irbesartan	7	340.64 ± 54.00^*∗∗*^	70.29 ± 39.08^*∗∗*##^

Data were presented as means ± SD.^*∗*^*P* < 0.05and ^*∗∗*^*P* < 0.01 versus the normal group; ^#^*P* < 0.05 and ^##^*P* < 0.01 versus the model group.

**Table 2:** Comparisons of TC, TG, HDL-C, and LDL-C in different groups after 8 weeks.

Group	*N*	TC (mmol/L)	TG (mmol/L)	LDL-C (mmol/L)	HDL-C (mmol/L)
Normal	7	1.63 ± 0.09	0.48 ± 0.11	0.48 ± 0.08	0.88 ± 0.07
Model	7	1.45 ± 0.16	0.82 ± 0.29^*∗*^	0.32 ± 0.08	0.83 ± 0.14
Keluoxin	7	1.36 ± 0.26	0.69 ± 0.33	0.29 ± 0.13	0.85 ± 0.17
Irbesartan	7	1.43 ± 0.19	0.71 ± 0.14	0.29 ± 0.16	0.96 ± 0.15

Data were presented as means ± SD.^*∗*^*P* < 0.05 and ^*∗∗*^*P* < 0.01 versus the normal group; ^#^*P* < 0.05 and ^##^*P* < 0.01 versus the model group.

**Table 3:** Comparisons of FPG and OGTT 2 h in different groups after 8 weeks.

Group	*N*	FPG (mmol/L)	OGTT 2 h (mmol/L)
Normal	7	6.34 ± 0.18	7.48 ± 0.1
Model	7	30.36 ± 1.67^*∗∗*^	30.14 ± 2.16^*∗∗*^
Keluoxin	7	26.74 ± 0.62^##^	28.72 ± 2.5
Irbesartan	7	31.60 ± 0.39	29.22 ± 2.93

Data were presented as means ± SD.^*∗*^*P* < 0.05 and ^*∗∗*^*P* < 0.01 versus the normal group; ^#^*P* < 0.05 and ^##^*P* < 0.01 versus the model group.

**Table 4:** Comparisons of LC3-l, LC3-ll, LC3-ll/LC3-l, p62, and nephrin in different groups after 8 weeks.

Group	*N*	LC3-l	LC3-ll	LC3-ll/LC3-l	p62	Nephrin
Normal	7	1.00 ± 0.00	1.00 ± 0.00	1.00 ± 0.00	1.00 ± 0.00	1.00 ± 0.00
Model	7	1.00 ± 0.22	1.55 ± 0.18^*∗∗*^	1.61 ± 0.33^*∗∗*^	1.58 ± 0.19^*∗∗*^	0.60 ± 0.08^*∗∗*^
Keluoxin	7	0.88 ± 0.15	1.28 ± 0.22^#^	1.17 ± 0.39^##^	1.21 ± 0.21^#^	0.94 ± 0.09^##^
Irbesartan	7	1.18 ± 0.37	1.30 ± 0.26^#^	1.49 ± 0.29^#^	1.19 ± 0.18^##^	0.86 ± 0.15^##^

Data were presented as means ± SD.^*∗*^*P* < 0.05 and ^*∗∗*^*P* < 0.01 versus the normal group; ^#^*P* < 0.05 and ^##^*P* < 0.01 versus the model group.

## Data Availability

The data used to support the findings of this study are included within the article.

## References

[1] Elkazzaz S. K., Khodeer D. M., El Fayoumi H. M., Moustafa Y. M. (2021). Role of sodium glucose cotransporter type 2 inhibitors dapagliflozin on diabetic nephropathy in rats; Inflammation, angiogenesis and apoptosis. *Life Sciences*.

[2] Nie Y., Fu C., Zhang H. (2020). Celastrol slows the progression of early diabetic nephropathy in rats via the PI3K/AKT pathway. *BMC complementary medicine and therapies*.

[3] Luk A. O. Y., Hui E. M. T., Sin M.-C. (2017). Declining trends of cardiovascular-renal complications and mortality in type 2 diabetes: the Hong Kong diabetes database. *Diabetes Care*.

[4] Wang X., Gao L., Lin H. (2018). Mangiferin prevents diabetic nephropathy progression and protects podocyte function via autophagy in diabetic rat glomeruli. *European Journal of Pharmacology*.

[5] Nagata M. (2016). Podocyte injury and its consequences. *Kidney International*.

[6] Shakeel M. (2015). Recent advances in understanding the role of oxidative stress in diabetic neuropathy. *Diabetes & Metabolic Syndrome: Clinical Research Reviews*.

[7] Ding Y., Choi M. E. (2015). Autophagy in diabetic nephropathy. *Journal of Endocrinology*.

[8] Parzych K. R., Klionsky D. J. (2014). An overview of autophagy: morphology, mechanism, and regulation. *Antioxidants and Redox Signaling*.

[9] Shi Y., Gao Y., Wang T. (2020). Ginsenoside Rg1 alleviates podocyte EMT passage by regulating AKT/GSK3 *β*/*β*-Catenin pathway by restoring autophagic activity. *Evidence-based Complementary and Alternative Medicine*.

[10] Li Y., Pan Y., Cao S. (2021). Podocyte EGFR inhibits autophagy through upregulation of rubicon in type 2 diabetic nephropathy. *Diabetes*.

[11] Xin W., Li Z., Xu Y. (2016). Autophagy protects human podocytes from high glucose-induced injury by preventing insulin resistance. *Metabolism*.

[12] Takabatake Y., Kimura T., Takahashi A., Isaka Y. (2014). Autophagy and the kidney: health and disease. *Nephrology Dialysis Transplantation*.

[13] Doria A., Gatto M., Punzi L. (2013). Autophagy in human health and disease. *New England Journal of Medicine*.

[14] Xu Y., Liu L., Xin W. (2015). The renoprotective role of autophagy activation in proximal tubular epithelial cells in diabetic nephropathy. *Journal of Diabetes and Its Complications*.

[15] Kume S., Maegawa H. (2020). Lipotoxicity, nutrient-sensing signals, and autophagy in diabetic nephropathy. *JMA Journal*.

[16] Wu F., Li S., Zhang N. (2018). Hispidulin alleviates high-glucose-induced podocyte injury by regulating protective autophagy. *Biomedicine & Pharmacotherapy*.

[17] Kim H., Dusabimana T., Kim S. R. (2018). Supplementation of abelmoschus manihot ameliorates diabetic nephropathy and hepatic steatosis by activating autophagy in mice. *Nutrients*.

[18] Xiao Y., Liu Y., Lai Z. (2021). An integrated network pharmacology and transcriptomic method to explore the mechanism of the total rhizoma coptidis alkaloids in improving diabetic nephropathy. *Journal of Ethnopharmacology*.

[19] Tu Q., Li Y., Jin J., Jiang X., Ren Y., He Q. (2019). Curcumin alleviates diabetic nephropathy via inhibiting podocyte mesenchymal transdifferentiation and inducing autophagy in rats and MPC5 cells. *Pharmaceutical Biology*.

[20] Liu Y., Liu W., Zhang Z. (2021). Yishen capsule promotes podocyte autophagy through regulating SIRT1/NF-*κ*B signaling pathway to improve diabetic nephropathy. *Renal Failure*.

[21] Wang H., Cui H., Lin L. (2019). The effects of a hirudin/liposome complex on a diabetic nephropathy rat model. *BMC Complementary and Alternative Medicine*.

[22] Zhang J., Xie X., Li C., Fu P. (2009). Systematic review of the renal protective effect of Astragalus membranaceus (root) on diabetic nephropathy in animal models. *Journal of Ethnopharmacology*.

[23] Kim J., Moon E., Kwon S. (2014). Effect of Astragalus membranaceus extract on diabetic nephropathy. *Endocrinology, Diabetes & Metabolism Case Reports*.

[24] Jing D., Bai H., Yin S. (2017). Renoprotective effects of emodin against diabetic nephropathy in rat models are mediated via PI3K/Akt/GSK-3beta and Bax/caspase-3 signaling pathways. *Experimental and Therapeutic Medicine*.

[25] Pang X., Zhang Y, Peng Z, Shi X, Han J, Xing Y (2020). Hirudin reduces nephropathy microangiopathy in STZ-induced diabetes rats by inhibiting endothelial cell migration and angiogenesis. *Life Sciences*.

[26] Guo M. F., Dai Y. J., Gao J. R., Chen P. J. (2020). Uncovering the mechanism of Astragalus membranaceus in the treatment of diabetic nephropathy based on network pharmacology. *Journal of diabetes research*.

[27] Wang F. L., Wang Y. H., Han L. (2018). Renoprotective effect of Yiqi Yangyin Huayu tongluo formula against diabetic nephropathy in diabetic rats. *Evidence-based Complementary and Alternative Medicine: ECAM*.

[28] Wei T.-T., Yang L.-T., Guo F. (2021). Activation of GPR120 in podocytes ameliorates kidney fibrosis and inflammation in diabetic nephropathy. *Acta Pharmacologica Sinica*.

[29] Zhang X., Zhang L., Chen Z. (2021). Exogenous spermine attenuates diabetic kidney injury in rats by inhibiting AMPK/mTOR signaling pathway. *International Journal of Molecular Medicine*.

[30] Zhang Y., Fukusumi Y., Kayaba M., Nakamura T., Sakamoto R., Ashizawa N. (2021). Xanthine oxidoreductase inhibitor topiroxostat ameliorates podocyte injury by inhibiting the reduction of nephrin and podoplanin. *Nefrologia*.

[31] Dai H., Liu Q., Liu B. (2017). Research progress on mechanism of podocyte depletion in diabetic nephropathy. *Journal of diabetes research*.

[32] Kawanami D., Matoba K., Utsunomiya K. (2016). Signaling pathways in diabetic nephropathy. *Histology & Histopathology*.

[33] Liu W. J., Gan Y., Huang W. F. (2019). Lysosome restoration to activate podocyte autophagy: a new therapeutic strategy for diabetic kidney disease. *Cell Death & Disease*.

[34] Kume S., Thomas M. C., Koya D. (2012). Nutrient sensing, autophagy, and diabetic nephropathy. *Diabetes*.

[35] Lenoir O., Jasiek M., Hénique C. (2015). Endothelial cell and podocyte autophagy synergistically protect from diabetes-induced glomerulosclerosis. *Autophagy*.

[36] Wu Y., Wang Y., Zhang J. (2021). Early-onset of type 2 diabetes mellitus is a risk factor for diabetic nephropathy progression: a biopsy-based study. *Aging*.

[37] Yasuda-Yamahara M., Kume S., Tagawa A., Maegawa H., Uzu T. (2015). Emerging role of podocyte autophagy in the progression of diabetic nephropathy. *Autophagy*.

[38] Armelloni S., Corbelli A., Giardino L. (2014). Podocytes: recent biomolecular developments. *Biomolecular Concepts*.

[39] Yoshii S. R., Mizushima N. (2017). Monitoring and measuring autophagy. *International Journal of Molecular Sciences*.

[40] Shen H.-M., Mizushima N. (2014). At the end of the autophagic road: an emerging understanding of lysosomal functions in autophagy. *Trends in Biochemical Sciences*.

[41] Liu W. J., Xu B.-H., Ye L. (2015). Urinary proteins induce lysosomal membrane permeabilization and lysosomal dysfunction in renal tubular epithelial cells. *American Journal of Physiology-Renal Physiology*.

[42] Ma T., Zhu J., Chen X., Zha D., Singhal P. C., Ding G. (2013). High glucose induces autophagy in podocytes. *Experimental Cell Research*.

